RETRACTED

# Diagnosis and Analysis of Transabdominal and Intracavitary Ultrasound in Gynecological Acute Abdomen

**DOI:** 10.1155/2021/9508838

**Published:** 2021-12-29

**Authors:** Huali Yang, Renying Wang, Liangchao Zhao, Jinhua Ye, Nengping Li, Lei Kong

**Affiliations:** ^1^Department of Obstetrics and Gynecology, Ruijin Hospital, School of Medicine, Shanghai Jiaotong University, Shanghai 201821, China; ^2^Department of Emergency, Ruijin Hospital, School of Medicine, Shanghai Jiaotong University, Shanghai 201821, China; ^3^Department of General Surgery, Ruijin Hospital, School of Medicine, Shanghai Jiaotong University, Shanghai 201821, China

## Abstract

In order to explore the effective diagnosis method of gynecological acute abdomen, this paper takes hospital gynecological acute abdomen patients as samples and selects gynecological acute abdomen patients admitted to the hospital to be included in this study. They are divided into transabdominal ultrasound group, intracavitary ultrasound group, and combined group. Moreover, this paper uses mathematical statistics to carry out sample statistics. The statistical data mainly include ectopic pregnancy, torsion of ovarian tumor pedicle, acute suppurative salpingitis, torsion of fallopian tube, hemorrhagic salpingitis, acute pelvic inflammatory disease, rupture of corpus luteum cyst, and diagnosis accuracy rate. In addition, this paper compares the diagnostic accuracy of the abdominal ultrasound group, the intracavitary ultrasound group, and the combined group. The experimental research shows that the combined ultrasound diagnosis method can effectively improve the accuracy of the diagnosis of gynecological acute abdomen.

## 1. Introduction

The incidence of acute abdomen in clinical gynecology is relatively high. As a common disease, patients with severe and sudden abdominal pain are the typical manifestations. The disease progresses relatively quickly, and the etiology and diagnosis are relatively complicated. If targeted diagnosis and intervention cannot be carried out effectively, the prognosis may be relatively poor, and severe cases may even threaten the life of the patient. As a result, rapid clinical diagnosis is critical. Additionally, individuals with gynecological acute abdomen have fast illness development, a convoluted etiology, and an abrupt beginning. Due to the fact that the majority of patients experience significant stomach pain and other symptoms, it is simple to have an effect on everyday life. If the appropriate diagnosis and therapy are not provided in a timely manner, the patient may lose out on the best treatment option, which might have catastrophic repercussions [1]. The benefits of ultrasound examination are ease of use, high diagnostic accuracy, and cheap cost. Abdominal ultrasonography and transvaginal ultrasound are the most often utilised procedures in gynecological acute abdomen. The content and size of the lesion may be monitored constantly, in real time, and dynamically, providing a foundation for the design of treatment programmes.

RETRACTED

Gynecologic acute abdomen may affect women of any age range, with the reproductive age group being the most prevalent. There have also been reports of kid patients [2] only in situations of ovarian tumor torsion. Ectopic pregnancy, ruptured corpus luteum, torsion of ovarian cyst pedicle, and acute pelvic inflammatory disease are the most frequent gynecological causes of acute abdomen. Ectopic pregnancy and acute pelvic inflammatory disease are the most common gynecological causes of acute abdomen. Ectopic pregnancy is the leading cause of mortality among women in their first trimester. Historically, the incidence rate was about 1%. Over the last 15 years, the global incidence rate has been increasing [3]. The prevalence of acute pelvic inflammatory illness is also increasing, and it has been found to be the most common cause of gynecological acute abdomen and the primary cause of tubal infertility. Due to the quick start of gynecological acute abdomen, a variety of illnesses may occur, and gynecologists are necessary to establish an accurate diagnosis and treat the patient promptly. In addition, when difficult problems are encountered, multidisciplinary consultation and collaboration are required to improve the accuracy of diagnosis. Timely and appropriate diagnosis and treatment measures are very important to reduce the occurrence of complications and sequelae. The advent of laparoscopy and its application in gynecological clinics has had a huge impact on the development of gynecological surgery. Laparoscopy is the gold standard for diagnosis of certain diseases such as endometriosis, pelvic, and abdominal adhesions. Moreover, it provides the possibility of early diagnosis and treatment of gynecological acute abdomen such as ectopic pregnancy, ovarian cyst torsion, ruptured corpus luteum, acute pelvic inflammatory disease, and pelvic abscess.

Intrauterine diseases include endometrial polyps, uterine submucosal fibroids, endometrial hyperplasia, endometrial cancer, IUD displacement, and uterine mediastinum. Numerous clinical signs exist, including vaginal bleeding irregularities, atypical menstruation, anemia, stomach discomfort, and irregular discharge. It may induce infertility, recurrent miscarriage, and other reproductive problems in women of childbearing age, posing a substantial danger to their reproductive prognosis and imposing significant social, psychological, and economic difficulties. Patients with suspected intrauterine lesions often receive a transvaginal two-dimensional ultrasound first. Further hysteroscopy is required for people who have concerns following a transvaginal two-dimensional ultrasound examination. With the advancement of hysteroscopy in recent years, the detection rate of intrauterine illnesses has risen year after year. Despite the fact that hysteroscopy is a minimally invasive procedure, it is nonetheless an invasive procedure with its own set of contraindications. Furthermore, it exposes the patient to infection, vasovagal syndrome, and uterine perforation, all of which have drawbacks. Furthermore, hysteroscopy requires specialised equipment and operating doctors, as well as being very costly, making it unsuitable for first screening in outpatient clinics. As a result, it is critical to develop a technique for doing an initial outpatient assessment that is relatively straightforward, noninvasive, affordable, and highly diagnostic.

RETRACTED

This article analyzes the diagnosis of gynecological acute abdomen by transabdominal and intracavitary ultrasound, combines data analysis to explore reliable diagnostic methods, and improves the diagnostic effect of gynecological acute abdomen.

## 2. Related Work

Gynecological acute abdomen is a kind of acute gynecological disease that is common clinically. Not only is it exceedingly abrupt but it also advances at a breakneck pace and is highly dangerous. Following the general onset, the patient's organs, retroperitoneal tissues, pelvic cavity, and abdominal cavity will show apparent pathological alterations, including acute lower abdominal discomfort, internal and external bleeding, and other symptoms, as well as systemic responses. If not addressed promptly, it may risk the patient's life [4]. Based on this, after clinical admission, it is necessary to determine the patient's specific type of acute abdomen in the shortest time and give a targeted treatment plan. However, the clinical manifestations of gynecological acute abdomen are not typical and specific. Therefore, in the actual clinical diagnosis work, the difficulty is relatively high; the probability of clinical missed diagnosis and misdiagnosis is high; it is easy to delay the patient's condition, affect the patient's prognosis, and even cause serious adverse consequences [5]. Therefore, there is an urgent need to find a scientific and efficient method for accurate diagnosis in clinic. In recent years, as China's medical technology has advanced, ultrasound technology has gotten more sophisticated. It not only speeds up the time-consuming diagnosis of gynecological acute abdomen but also increases clinical detection rates, provides a scientific and trustworthy reference for doctors to appropriately appraise the patient's status, and reduces the danger of accidents. At present, there are two widely used clinical ultrasound diagnostic techniques, namely, abdominal ultrasound and vaginal ultrasound. No matter which method of diagnosis, each has its own advantages and certain limitations. Therefore, many clinical scholars have proposed a joint diagnosis method [6].

RETRACTED

Ectopic pregnancy is the most common disease in gynecological emergencies, among which tubal pregnancy accounts for 95% to 98%. Laparoscopic treatment of tubal pregnancy is one of the earliest and most mature operations in laparoscopic gynecological surgery. Surgical methods can be divided into radical surgery and conservative surgery. The choice of surgical procedure mainly depends on factors such as the age of the patient, whether there are fertility requirements, and the degree of damage to the fallopian tubes of pregnancy [7]; major surgery may be conducted on women who have had children and are no longer pregnant. Conservative surgery is appropriate for women who have not given birth and for young women who need fallopian tube preservation and must adhere to the following: ① Pregnancy is located in the umbrella, ampulla, or isthmus of the fallopian tube, while the interstitial pregnancy generally does not choose conservative surgery. ② Tubal pregnancy is unruptured, or although it has been ruptured, the rupture is small. ③ The diameter of the tubal pregnancy lesion is less than 5 cm, the internal bleeding is not much, and the patient's vital signs are stable. ④ No pelvic or intra-abdominal infection [8]. To avoid clamping the mucous membrane of the fallopian tube, causing unnecessary damage and difficulty in hemostasis, conservative surgery requires the surgeon to have proficient surgical skills and a meticulous work style, electrocoagulation cut the affected area of the fallopian tube serosa, grasping forceps to remove pregnancy products and blood clots, and grasping forceps to remove pregnancy products and blood clots [9]. Conservative surgery for fallopian tube hemostasis may be challenging, although local compression, no fallopian tube injury using a fallopian tube clamp, and local spraying of “restophemostasis” and other hemostatic techniques are all options [10]. Conservative surgery may be difficult at times to fully remove the trophoblast cells in the fallopian tube, which can lead to ectopic pregnancy, fallopian tube rupture, internal bleeding, and reoperation. As a result, variations in blood *β*-HCG should be monitored following a conservative fallopian tube procedure, and MTX should be utilised if the *β*-HCG goes below 20% within one week of the operation [11]. Conservative surgery should not be chosen for keratointerstitial pregnancy owing to the abundant blood vessels and difficulties in hemostasis, according to the literature [12], although salpingectomy on the afflicted side is possible. Although there have been several publications in the literature demonstrating laparoscopy's evident benefits in the treatment of ectopic pregnancy, its use to rescue shock-type tubal pregnancy remains contentious in China. According to the research [13], rupture of an ectopic pregnancy with significant bleeding and active bleeding in the lesion does not exclude laparoscopic surgery. As long as the operation is handled properly, the operation can be successfully completed. A large number of foreign documents show that laparoscopic surgery is safe and effective in the treatment of hypovolemic shock ectopic pregnancy [14]. The literature [15] believes that under the premise of effective antishock treatment, laparoscopic surgery is the first choice for the treatment of shock-type tubal pregnancy. Moreover, compared with open surgery, laparoscopic surgery for ectopic pregnancy has less bleeding, shorter hospital stay, higher pregnancy rate after surgery, and lower risk of pregnancy and reectopic pregnancy in the short term after surgery.

RETRACTED

The fallopian tube function is impaired by acute pelvic inflammatory illness, particularly the development of inflammatory masses such as fallopian tube abscess and fallopian tube ovarian abscess. According to the literature [16], the incidence of acute pelvic inflammatory illness is on the rise, and it is the most common gynecological acute abdomen, as well as the leading cause of tubal infertility. As a result, it is critical to diagnose and treat acute pelvic inflammatory illness as soon as possible. Acute pelvic inflammatory illness was formerly thought to be a contraindication to laparoscopic surgery. The biggest fear was that laparoscopic surgery and intraoperative washing might cause inflammation to spread due to the high hips and low head. It is no longer mentioned as a contraindication for laparoscopic surgery but rather as an indication, after many years of clinical experience. According to the literature [17], the coincidence rate between PID identified using stringent clinical diagnostic criteria and PID diagnosed using laparoscopy is only 65%, and all domestic and international publications agree that laparoscopic diagnosis is the gold standard for pelvic inflammatory disease. Because to the tiny incision, laparoscopy has a lower risk of wound infection. Avoid infections such as acute pelvic inflammatory illness, pelvic abscess, and open surgical wounds. Laparoscopic surgery is more costly, intrusive, and susceptible to the surgeon's subjective constraints. As a result, the question of when to select laparoscopic surgery for acute pelvic inflammatory disease is a hot topic right now. According to the research [18], patients with persistent masses after 24–72 hours of medication therapy or one or two weeks of antibiotic treatment should be considered for pelvic inflammatory disease surgery. Surgery should also be considered aggressively in individuals with an uncertain clinical diagnosis, substantial pelvic masses, recurring episodes, or reproductive needs. Literature [19] studied the fibrous adhesions in the pelvic cavity of PID patients and found that these fibrous cords contain a considerable amount of bacteria. If they are not thoroughly cleaned, it is easy to induce pelvic inflammation and pelvic abscess again. According to reports by Jin Liping and others, it was found that the adhesions between the tissues in the acute phase of PID are relatively loose and easy to separate, and it is confirmed that within 1 week of the infection, the inflammatory exudates on the surface of the organs have not been organized, and the adhesions are soft and not formed. The sturdy fiber band is conducive to the operation. If you are fully prepared and operated carefully during the operation, the operation is very safe.

RETRACTED

## 3. Method

This article selects gynecological acute abdomen patients admitted to the hospital to be included in this study. They are divided into transabdominal ultrasound group, intracavitary ultrasound group, and combined group. All patients were accompanied by symptoms such as abdominal pain, fever, and vaginal bleeding of varying degrees. They were informed and voluntarily cooperated with this study, all signed a consent form, and the hospital ethics committee approved the development of the study. There was no significant difference between the two groups of patients in general data such as age, gender, marital status, and statistical significance (*P* > 0.05), which is comparable.

Transabdominal ultrasonography was utilised for examination, and colour Doppler ultrasound was employed in the transabdominal ultrasound group. Patients are advised to drink lots of water to fill their bladders before to the test. The patient is positioned in a supine posture with the transabdominal probe frequency set at 3.55.0 MHz. The probe is inserted into the patient's belly to check for masses, gestational sacs, pelvic fluid, and uterine wall echo within and outside the uterine cavity, as well as measure and record aberrant data. The findings of transabdominal ultrasonography are compared to the results of pathological diagnosis, and the rate of transabdominal ultrasonography results that correspond is computed.

RETRACTED

Transvaginal and transabdominal ultrasonography are used to assess the mixed group. The transabdominal ultrasound group uses the same procedures and tools as the transabdominal ultrasound group. The patient was ordered to empty his bladder after the transabdominal ultrasound examination, and he assumed the lithotomy position, elevated his buttocks, and exposed his perineum. The probe is coated with couplant and wrapped with a clean disposable condom. The frequency of the probe is set at 5.0–8.0 MHz, enters the vaginal vault gently via the patient's vagina, and does scanning examinations of various areas using rotating, tilting, swinging, and other ways. Additionally, it examines the patient's ovaries and uterus for size and form, as well as the echo within the uterus and the endometrium, as well as the appendages on both sides and the pelvic wall, both inside and outside the uterine cavity. When necessary, we need to press the patient through the abdomen with hands to bring the probe closer to the examination area, display a clear image, and observe whether there are lumps and pelvic fluid. If a mass is found, it is observed whether there is a gestational sac inside it. If pelvic effusion is found, data such as effusion depth and blood flow characteristics should be recorded. The results of vaginal combined transabdominal ultrasonography were compared with the results of pathological diagnosis. The coincidence rate of vaginal combined transabdominal ultrasonography was calculated.

The statistical data in this paper mainly include ectopic pregnancy, torsion of ovarian tumor pedicle, acute suppurative salpingitis, torsion of fallopian tube, hemorrhagic salpingitis, acute pelvic inflammatory disease, rupture of corpus luteum cyst, and diagnosis accuracy rate.

## 4. Result

This paper counts the diagnostic accuracy rates of ectopic pregnancy, torsion of ovarian tumor pedicle, acute suppurative salpingitis, torsion of fallopian tube, hemorrhagic salpingitis, acute pelvic inflammatory disease, and rupture of corpus luteum cyst. The results obtained are shown in Tables 1–7.

## 5. Analysis and Discussion

Gynecological acute abdomen is a category of acute abdomen, which refers to various types of acute abdomen that are specific to women, including ectopic pregnancy, torsion of ovarian cyst pedicle, rupture of corpus luteum cyst, and acute pelvic inflammatory disease. Its clinical features are similar to other acute abdomen, all manifested as sudden transabdominal pain, which may be accompanied by progressive aggravation. At the beginning of the onset of some patients, it turned out to be dull pain in the area of transabdominal patients, with mild pain and paroxysmal pain. If it is not treated in time, it can cause systemic inflammation. The causes of gynecological acute abdomen are more varied, including surgical complications, infection, and concomitant disorders. For instance, insufficient treatment of chronic pelvic inflammatory illness might result in the development of other adjacent tissues. For acute abdomen produced by acute abdomen in patients with noticeable pain and impact, it is often recommended to initiate treatment promptly to prevent further development of the situation, which also places increased demands on the diagnostic technology for different gynecological acute abdomen. Gynecological acute abdomen refers to severe abdominal pain caused by gynecological diseases. At present, common acute abdomen in gynecology mainly includes ectopic pregnancy, rupture of the corpus luteum, torsion of ovarian cyst pedicle, rupture of ovarian cyst, adenomyosis, and gynecological inflammatory diseases such as acute pelvic inflammatory disease. Ectopic pregnancy is also called ectopic pregnancy. It means that the patient is pregnant, but the pregnant part is not in the uterine cavity but in a position outside the uterine cavity. The conceived ovum is implanted in the fallopian tube but not in the uterus. Menopause is the primary symptom, followed by stomach discomfort, a little quantity of vaginal bleeding, and a sensation of swelling in the anus. Additionally, some people have no apparent history of menopause, which is evidenced by intermittent vaginal bleeding. Pregnancy is not possible via the fallopian tube. With increasing gestational age, pregnant mass rupture, bleeding, and even death may ensue. Once ectopic pregnancy breaks down, it will lead to intra-abdominal bleeding and blood pressure drop, and finally hemorrhagic shock may occur. The situation is urgent, and urgent surgery is required. Rupture of the corpus luteum generally occurs during the second part of the menstrual cycle. Patients with torsion of the pedicle of ovarian cysts have a history of ovarian cysts, which frequently develop following a change in posture and cause abrupt lower abdominal discomfort. The symptoms are similar to those of an ectopic pregnancy, but the discomfort is less severe and may be addressed without surgery. Patients with twisted ovarian cyst pedicles have previously had ovarian cysts. Sudden lower transabdominal or lateral transabdominal pain after vigorous activity or position changes; the pain might be increased or reduced with a change of posture, and it is sometimes difficult to differentiate from appendicitis. Surgery should be undertaken as soon as feasible when the diagnosis has been established. Multiple disorders, complicated circumstances, fast onset, and rapid changes characterise gynecological acute abdomen. If the nature and cause of the sickness are not identified quickly, the condition may deteriorate, making treatment more difficult and perhaps putting the patient's life in jeopardy. Patients have received positive news as a result of the advancement of ultrasound technology. Patients choose ultrasound examination technology because of its noninvasiveness, ease of operation, cost savings, and broad application range, and it is easily accepted by patients. Transabdominal ultrasonography scans a vast area and depicts the pathology of the patient clearly.

RETRACTED

At present, the diagnosis of gynecological acute abdomen is mainly based on imaging examination, and ultrasound examination is one of the core technologies, including transabdominal ultrasound and transvaginal ultrasound. Transabdominal ultrasound is a widely used ultrasound examination technique. The principle of this technology is to introduce sound waves into the human body, and the interface reflection between different tissues can produce echo and then return to the probe. The returning sound waves cause the unit of the probe to oscillate and convert the oscillations into electrical pulses. The probe transmits the pulse to the ultrasonic host, which converts it to a digital picture for analysis of the lesion information in the tissue, determining the presence of a lesion, its area, category, and severity. The disadvantage of this technology is that it can accurately screen small lesions and is affected by multiple dynamic factors, so its applicability is limited. For example, when the patient's body is relatively obese, the fat layer will affect the scientificity of the imaging results, causing difficulties in diagnosis and identification. The transvaginal combined transabdominal ultrasound examination is the same in principle as the transabdominal ultrasound; that is, it uses the introduction of sound waves and echo collection for imaging. Compared with a single transabdominal ultrasound diagnosis, transvaginal ultrasound diagnosis can avoid the influence of the patient's transabdominal fat layer and abdominal intestinal gas and obtain a clearer impact assessment of the condition. At the same time, the influence of different angles is also more three-dimensional, which helps to realize the effective detection and identification of the disease. For example, the clarity of transabdominal ultrasound pictures is inadequate for the assessment of bilateral ovarian cysts; it is difficult to collect precise and sensitive indicators, and the impact of inspection and differential diagnosis is impossible to ensure. Following transvaginal and transabdominal ultrasonography, the pictures are overlaid to produce clear and sensitive data that may be used to ensure diagnostic specificity. Evident ultrasound echo enhancement regions and edge echo enhancement features may be noticed in the patient's imaging data, which are comparable in specificity to pure transabdominal ultrasound imaging. It does, however, have more clarity and sensitivity, which makes it more useful for illness detection and differential diagnosis. Transvaginal and transabdominal ultrasonography may be used together to acquire reliable information about the patient's condition. Various types of inflammation that occur in different places may be recognised, as can different diseases that occur in the same place. For example, under the effect of ultrasonography, hyperplastic lesions and inflammatory lesions might detect modest echoes, and the echo augmentation is not noticeable when compared to the surroundings. The echo amplification of inflammatory lesions is more noticeable, and its intensity variations with surrounding tissues are compared, allowing not only for the diagnosis of the illness's location but also for the comprehensive identification of the disease kind and a better inspection impact. It is worth noting that when compared to MRI, CT, and pathological examination, ultrasound diagnosis is very effective and economical and hence should be widely promoted. However, there are still issues with clarity, sensitivity, and specificity. Some illnesses have a poor detection rate, and differential diagnostic accuracy still has to be improved. In conclusion, when compared to transabdominal ultrasound, transvaginal mixed with transabdominal ultrasound can successfully identify gynecological acute abdomen, has a high detection rate for various illnesses, and has a higher specificity and sensitivity. Patients with acute abdomen in gynecology may be identified using transvaginal mixed with transabdominal ultrasound in the follow-up work, and different illnesses can be properly discovered, and symptomatic therapy can be offered to assure the patients' prognosis.

RETRACTED

## Figures and Tables

**Table 1:** Accuracy of diagnosis of ectopic pregnancy.

Number	Transabdominal ultrasound	Intracavitary ultrasound	Combined ultrasound	Number	Transabdominal ultrasound	Intracavitary ultrasound	Combined ultrasound
1	58.90	73.16	93.30	16	69.96	87.61	93.50
2	69.59	71.43	91.14	17	78.10	79.63	92.90
3	65.89	83.97	97.38	18	68.80	72.96	98.41
4	68.28	77.24	95.11	19	88.18	67.76	93.88
5	61.64	89.62	95.15	20	71.46	88.45	96.22
6	73.67	91.75	95.57	21	59.97	84.64	95.27
7	58.42	79.77	98.71	22	61.33	76.45	97.39
8	72.18	67.95	98.68	23	70.87	85.16	97.48
9	66.09	75.21	94.85	24	70.62	72.89	97.93
10	71.67	85.61	91.95	25	60.99	80.42	93.50
11	87.29	72.70	95.56	26	87.62	74.63	93.91
12	63.27	83.44	91.20	27	70.38	69.60	97.22
13	74.96	76.87	92.12	28	70.19	84.13	96.16
14	74.60	82.33	98.19	29	81.97	74.91	97.93
15	66.28	90.47	96.93	30	64.34	87.58	94.02

**Table 2:** Accuracy of diagnosis of ovarian tumor pedicle torsion.

Number	Transabdominal ultrasound	Intracavitary ultrasound	Combined ultrasound	Number	Transabdominal ultrasound	Intracavitary ultrasound	Combined ultrasound
1	68.04	90.71	92.32	16	86.02	76.48	98.81
2	85.01	69.63	95.83	17	73.27	88.13	91.29
3	81.94	74.99	94.71	18	60.43	91.61	91.78
4	88.72	88.18	96.24	19	80.34	84.74	98.20
5	79.78	81.52	98.79	20	61.77	83.73	91.73
6	58.66	82.80	97.87	21	60.20	90.57	91.43
7	76.76	78.95	92.62	22	60.16	76.98	93.63
8	70.09	89.86	94.77	23	85.74	68.79	95.66
9	70.68	76.35	98.83	24	73.35	75.00	96.63
10	65.51	87.14	97.09	25	71.05	67.52	95.10
11	61.22	83.71	92.41	26	63.06	81.03	92.28
12	59.33	69.09	97.65	27	65.45	91.83	93.09
13	77.07	84.32	98.33	28	75.52	75.92	94.71
14	62.67	67.00	91.02	29	77.40	73.12	98.34
15	76.76	77.99	95.72	30	67.47	77.27	93.98

**Table 3:** Accuracy of diagnosis of acute suppurative salpingitis.

Number	Transabdominal ultrasound	Intracavitary ultrasound	Combined ultrasound	Number	Transabdominal ultrasound	Intracavitary ultrasound	Combined ultrasound
1	65.53	72.44	93.63	16	60.58	82.62	94.04
2	83.87	85.66	91.51	17	87.29	75.18	96.72
3	60.47	67.99	97.57	18	70.32	87.47	94.00
4	70.72	72.53	93.83	19	72.32	67.75	98.87
5	69.84	72.93	98.27	20	79.19	78.11	91.11
6	80.12	73.92	95.91	21	70.29	71.29	93.39
7	80.18	69.76	94.78	22	65.41	79.42	94.02
8	63.80	77.96	94.69	23	81.38	67.34	91.41
9	64.14	69.07	92.97	24	63.41	91.93	95.81
10	63.25	73.92	96.70	25	74.20	85.61	93.37
11	68.73	83.65	98.33	26	80.60	71.85	97.56
12	87.12	91.78	98.25	27	85.68	71.93	98.39
13	66.48	67.31	97.51	28	70.27	67.81	94.50
14	77.70	91.29	95.74	29	84.79	78.76	94.66
15	86.67	84.23	95.30	30	76.38	74.12	97.64

**Table 4:** Accuracy of diagnosis of fallopian tube torsion.

Number	Transabdominal ultrasound	Intracavitary ultrasound	Combined ultrasound	Number	Transabdominal ultrasound	Intracavitary ultrasound	Combined ultrasound
1	65.42	85.65	92.27	16	73.63	85.70	98.91
2	61.42	83.66	93.67	17	84.51	73.83	95.24
3	79.06	76.27	92.63	18	71.46	87.11	92.48
4	60.99	80.67	93.65	19	72.99	83.31	96.05
5	69.55	87.68	92.38	20	73.32	81.51	92.22
6	87.56	73.80	92.50	21	80.84	70.23	92.37
7	73.80	84.85	96.91	22	63.86	84.69	94.89
8	62.65	67.43	98.46	23	67.51	67.15	97.94
9	71.70	87.90	92.15	24	79.29	82.36	96.54
10	63.33	87.70	95.78	25	62.40	84.70	96.06
11	61.99	69.67	98.21	26	86.53	72.34	93.38
12	70.60	82.68	97.24	27	77.87	70.44	97.31
13	71.78	78.71	93.93	28	83.28	67.77	91.78
14	83.90	67.49	93.62	29	64.73	72.15	94.28
15	58.41	69.87	91.16	30	82.07	90.22	97.89

RETRACTED

**Table 5:** Accuracy of diagnosis of hemorrhagic salpingitis.

Number	Transabdominal ultrasound	Intracavitary ultrasound	Combined ultrasound	Number	Transabdominal ultrasound	Intracavitary ultrasound	Combined ultrasound
1	71.48	68.07	96.99	16	76.70	71.10	95.79
2	62.53	77.43	92.84	17	81.84	68.92	96.89
3	63.85	83.35	94.47	18	85.18	69.85	95.30
4	71.13	78.07	97.85	19	64.92	87.39	91.92
5	62.38	82.93	94.55	20	68.11	68.69	98.27
6	69.48	74.90	91.19	21	75.46	76.14	94.67
7	62.08	81.83	97.88	22	88.60	67.91	98.00
8	83.09	88.38	96.74	23	76.87	67.69	92.33
9	83.89	89.61	95.43	24	58.45	83.01	93.40
10	75.78	91.45	92.71	25	70.19	77.87	97.48
11	73.96	74.71	96.94	26	74.42	69.86	96.86
12	80.70	91.84	97.35	27	59.01	89.31	98.48
13	77.94	80.65	97.25	28	69.15	86.91	93.23
14	67.59	69.51	95.29	29	58.73	81.11	98.52
15	87.16	80.62	93.00	30	62.13	85.19	91.91

**Table 6:** Accuracy of diagnosis of acute pelvic inflammatory disease.

Number	Transabdominal ultrasound	Intracavitary ultrasound	Combined ultrasound	Number	Transabdominal ultrasound	Intracavitary ultrasound	Combined ultrasound
1	59.73	75.91	91.73	16	84.48	91.05	95.16
2	71.00	73.50	94.06	17	75.05	71.93	97.94
3	75.48	74.89	95.98	18	68.05	83.31	92.90
4	71.51	88.84	97.36	19	70.46	78.40	95.04
5	80.59	75.08	98.90	20	66.91	78.10	92.33
6	73.19	75.58	92.95	21	71.02	78.56	95.65
7	73.13	76.95	97.38	22	69.72	76.50	92.89
8	60.20	76.70	91.83	23	85.11	87.03	94.46
9	59.64	70.77	92.45	24	73.90	74.51	95.96
10	86.35	91.82	94.93	25	80.98	70.44	94.87
11	75.18	72.34	97.99	26	60.89	83.79	97.10
12	83.16	73.23	93.18	27	83.84	84.81	92.55
13	61.63	85.96	94.88	28	77.78	78.76	96.18
14	75.89	77.53	91.39	29	57.76	86.83	98.67
15	76.00	67.86	95.77	30	62.62	70.68	91.63

**Table 7:** Accuracy of diagnosis of ruptured ovarian corpus luteum cyst.

Number	Transabdominal ultrasound	Intracavitary ultrasound	Combined ultrasound	Number	Transabdominal ultrasound	Intracavitary ultrasound	Combined ultrasound
1	77.83	88.21	96.14	16	79.66	68.75	95.18
2	63.46	72.11	97.31	17	60.66	87.85	98.79
3	80.18	86.34	92.38	18	60.24	72.40	95.68
4	64.61	76.06	92.59	19	88.17	76.67	95.26
5	73.86	77.63	95.16	20	70.69	78.97	91.47
6	85.34	72.84	98.12	21	77.32	84.39	93.27
7	86.30	81.69	98.26	22	83.58	78.65	91.80
8	87.96	81.64	91.95	23	57.76	82.62	97.24
9	78.89	74.02	94.75	24	63.91	69.49	98.76
10	62.10	73.89	94.93	25	69.56	72.82	91.24
11	70.75	91.89	93.29	26	88.52	75.55	94.68
12	74.63	79.41	92.88	27	68.04	77.81	92.94
13	76.32	77.33	94.18	28	76.49	78.21	95.71
14	88.88	79.87	94.79	29	80.93	72.68	93.95
15	87.18	71.76	98.78	30	57.42	69.39	95.87

RETRACTED

## Data Availability

The data used to support the findings of this study are included within the article.
